# The Antioxidant and Starch Hydrolase Inhibitory Activity of Ten Spices in an* In Vitro* Model of Digestion: Bioaccessibility of Anthocyanins and Carotenoids

This article has been retracted.

**DOI:** 10.1155/2015/764238

**Published:** 2015-11-29

**Authors:** Nilakshi Jayawardena, Mindani I. Watawana, Ruchini T. Jayathilaka, Viduranga Y. Waisundara

**Affiliations:** Functional Food Product Development Project, National Institute of Fundamental Studies, Hantane Road, 20000 Kandy, Sri Lanka

## Abstract

The antioxidant and starch hydrolase inhibitory activities of cardamom, cloves, coriander, cumin seeds, curry leaves, fenugreek, mustard seeds, nutmeg, sweet cumin, and star anise extracts were investigated in an* in vitro* model of digestion mimicking the gastric and duodenal conditions. The total phenolic contents in all spice extracts had statistically significantly (*P* < 0.05) increased following both gastric and duodenal digestion. This was also in correlation with the antioxidant assays quantifying the water-soluble antioxidant capacity of the extracts. The lipophilic Oxygen Radical Absorbance Capacity assay did not indicate a statistically significant change in the values during any of the digestion phases. Statistically significant (*P* < 0.05) reductions in the anthocyanin contents were observed during the digestion phases in contrast to the carotenoid contents. With the exception of the cumin seed extract, none of the spice extracts showed statistically significant changes in the initial starch hydrolase enzyme inhibitory values prior to gastric and duodenal digestion. In conclusion, this study was able to prove that the 10 spices were a significant source of total phenolics, antioxidant, and starch hydrolase inhibitory activities.

## 1. Introduction

Antioxidant and starch hydrolase inhibitory activities are two of the most coveted mechanisms to which prevention of noncommunicable diseases such as cardiovascular disease (CVD), diabetes, and cancer is currently attributed. While antioxidants provide protection from cellular damage due to free radicals, starch hydrolase inhibitory activity is known to prevent the sudden release of glucose into the physiological system, thereby preventing the biochemical pathways which trigger the production of free radicals inside the mitochondria [1, 2]. Carotenoids and phenolic compounds have been identified as two major dietary antioxidants with both categories containing over hundred member compounds. Carotenoids are fat-soluble pigments, while phenolic compounds commonly exist as free, esterified, etherified, and insoluble-bound forms. The most abundant form of phenolic compounds is flavonoids, which are abundantly found in edible fruits, leafy vegetables, roots, tubers, bulbs, herbs, spices, and legumes [3, 4]. Other than antioxidant activity, certain flavonoids are known to possess the ability to modulate cellular enzyme activities—a trait which is responsible for the inhibition of starch hydrolases such as *α*-amylase and *α*-glucosidase [5]. Measurement of antioxidant and starch hydrolase inhibitory activities is well documented. Several chemical and biochemical assays have been utilized for the quantification of the total antioxidant capacity (TAC) of plant products [6]. In addition, with reference to phenolic compounds, a number of studies present a measure of the total polyphenol content of food products in order to draw comparisons with other similar products and to provide more detailed information about this subgroup of antioxidants [7, 8]. However, in this respect, a major obstacle in evaluating the role of individual food components in modifying disease risk is the scarcity of information on factors that influence their bioavailability and bioaccessibility [9].

Bioavailability is the degree to which a drug, nutrient, dietary supplement, or nutraceutical is available to the body. On the other hand, bioaccessibility is defined as the amount of a food constituent that is present in the gut, as a consequence of the release of this constituent from the solid food matrix, and may be able to pass through the intestinal barrier [10]. Several* in vitro* methods have been used to determine the bioaccessibility and bioavailability of individual antioxidant compounds in order to isolate those which remain stable and active throughout the digestion and absorption processes [5, 8, 9]. Only bioactive compounds released from the food matrix by the action of digestive enzymes present in pancreatic and duodenal digestion and bacterial microflora (large intestine) are bioaccessible in the gut and therefore potentially bioavailable. From this perspective, the amount of bioaccessible food antioxidants and other therapeutic compounds of interest may differ quantitatively and qualitatively from polyphenols included in food databases [11]. Given these conditions, the aim of this research was to quantify polyphenol contents, TAC, and starch hydrolase inhibitory activity of the acetone/water extracts of 10 commonly consumed spices and assess the stability of these parameters after the gastric and duodenal digestion phases in an* in vitro* model. Besides flavoring purposes, spices and herbs are known for their medical or antiseptic properties—characteristics which have been owed to the presence of immense amounts of antioxidant compounds [12]. In fact, the preservative effect of many spices and herbs suggests the presence of antioxidant and antimicrobial constituents [12, 13]. Special attention was rendered towards the analysis of anthocyanins which are abundantly present in the selected spices. Although flavonoids and phenolic acids are relatively more stable under the duodenal digestion conditions, anthocyanins are known to undergo ring fission during physiological digestion due to the varied pH conditions [14]. Selected carotenoids compounds are also quantified in order to provide a more holistic view on the effect of the digestion procedure on various types of antioxidant compounds.

## 2. Materials and Methods

All reagents, chemicals, and HPLC standards used for this study were purchased from Sigma Chemicals (St. Louis, MO, USA).

### 2.1. Preparation of Spice Powders and* In Vitro* Digestion Procedure

The following spices were chosen for the study based on their therapeutic properties, previous studies on antioxidant and starch hydrolase inhibitory properties as documented in the published literature [15–17]: cardamom (*Elettaria cardamomum*), cloves (*Syzygium aromaticum*), coriander (*Coriandrum sativum*), cumin seeds (*Cuminum cyminum*), curry leaves (*Murraya koenigii*), fenugreek (*Trigonella foenum*), mustard (*Brassica nigra*), nutmeg (*Myristica fragrans*), sweet cumin (*Pimpinella anisum*), and star anise (*Illicium verum*). Dried powders of the spices were obtained from the Ayurvedic Medicinal Hall in Kandy, Sri Lanka. The methodology by Wu et al. [18] was followed for the preparation of the herbal extracts using acetone/water/acetic acid (70 : 29.5 : 0.5). The* in vitro* digestion model was adapted from Ryan et al. [12]. In brief, the extracts of samples were transferred to clean amber bottles and mixed with saline (balanced salt solution) to create a final volume of 20 mL. The samples were acidified to pH 2.0 with 1 mL of a porcine pepsin preparation (0.04 g pepsin in 1 mL 0.1 M HCl) and incubated at 37°C in a shaking water bath at 3000 g for 1 h. After gastric digestion, 500 *μ*L of each sample was extracted and stored at −20°C. The pH was then increased to 5.3 with 0.9 M sodium bicarbonate followed by the addition of 200 *μ*L of bile salts glycodeoxycholate (0.04 g in 1 mL saline), taurodeoxycholate (0.025 g in 1 mL saline), and taurocholate (0.04 g in 1 mL saline) and 100 *μ*L of pancreatin (0.04 g in 500 *μ*L saline). The pH of each sample was increased to 7.4 with 1 M NaOH. Samples were incubated in a shaking water bath at 95 rpm at 37°C for 2 h to complete the intestinal phase of the* in vitro* digestion process. After the intestinal phase, 500 *μ*L of each sample was extracted and stored at −20°C. Digested samples were analyzed within 2 weeks.

### 2.2. Total Phenolic Content and Antioxidant Activity Assays

The total phenolic contents were determined according to Singleton et al. [17]. The values were expressed as *μ*g gallic acid equivalents per gram fresh weight (*μ*g GAE/g) of sample. Quantification of the water-soluble Oxygen Radical Absorbance Capacity (ORAC_FL_) was carried out according to the method by Prior et al. [19], while the lipophilic Oxygen Radical Absorbance Capacity (ORAC_oil_) was carried out according to the method by Hay et al. [20]. The DPPH method was conducted using the method by Brand-Williams et al. [21]. The FRAP assay was carried out as described by Benzie and Strain [22]. In addition, the antioxidant activities of the samples were analyzed by investigating their ability to scavenge the ABTS•+ using a methodology previously reported by Ozgen et al. [23]. All assays were carried out in 96-well plate format using the Synergy HTX multimode microplate reader and Gen5 software (Biotek, Winooski, VT, USA).

### 2.3. Assays of *α*-Amylase and *α*-Glucosidase Inhibitory Activities

The *α*-amylase inhibitory activity of the extracts was carried out according to the method by Liu et al. [24], while the *α*-glucosidase inhibitory activity was carried out according to the method by Koh et al. [25]. Both assays were carried out in 96-well plate format using the Synergy HTX multimode microplate reader and Gen5 software (Biotek, Winooski, VT, USA). Data were expressed as IC_50_ (mg/mL).

### 2.4. Total Monomeric Anthocyanin Pigment Content and High Performance Liquid Chromatography (HPLC) Determination of the Individual Anthocyanin Compounds

The AOAC official method 2005.02 [26] was carried out to quantify the total monomeric anthocyanin pigment content. The values were expressed as mg cyanidin-3-glucoside equivalents per gram wet weight of spice. The quantities of the individual anthocyanin compounds cyanidin-3-O-galactoside (C3Ga), cyanidin-3-O-glucoside (C3Gl), cyanidin-3-O-arabinoside (C3Ar), delphinidin-3-glucoside (D3Gl), peonidin-3-O-galactoside (P3Ga), and peonidin-3-O-arabinoside (P3Ar) were measured according to the method by Brown and Shipley [27]. Ten milliliters of solvent was centrifuged at 3000 g for 10 min. A volume of 1000 *μ*L of the extracts were diluted with 500 *μ*L of the extraction solvent (acetone/water/acetic acid, 70 : 29.5 : 0.5). Approximately 1 mL of solution was filtered through a 0.45 *μ*m nylon filter into an amber HPLC vial. The quantities of the individual anthocyanin compounds were quantified in the extracts using standards. A Shimadzu (Kyoto, Japan) HPLC system equipped with a diode array detector (SPDM10Avp) and a Phenomenex Luna C-18(2) column (4.6 mm i.d. × 25 cm, 5 *μ*m) was used for the quantification.

### 2.5. HPLC Determination of Carotenoids

Sample extraction and HPLC analysis for carotenoids (neoxanthin, violaxanthin, lutein, zeaxanthin, *α*-carotene, and *β*-carotene) were carried out according to the internal standard (IS) method by Lee et al. [28]. The Shimadzu (Kyoto, Japan) HPLC system equipped with a Phenomenex Luna C-18(2) column (4.6 mm i.d. × 25 cm, 5 *μ*m) was used for the quantification having cross-linked end-capping with diode array (SPDM10Avp) detection. At least triplicate extractions were performed for each sample. IS solution was weekly prepared according to the method by Lee et al. [28]. For calibration, 100 *μ*L of the IS solution was mixed with 100 *μ*L of standard mixtures of various concentrations. Stock solutions of each standard were prepared individually with relevant solvents as described by Lee et al. [29].

### 2.6. Statistical Analysis

All results are presented as mean ± standard error mean (SEM). For comparisons, data was analyzed by ANOVA and Tukey's multiple comparison test (SPSS, version 17). A probability of 5% or less was accepted as statistically significant.

## 3. Results and Discussion

### 3.1. Total Phenolic Contents, Antioxidant Activities, Anthocyanin, and Carotenoid Contents

The total phenolic contents are shown in Table 1. Cloves had the highest total phenolic content (22.83 ± 0.20 mg GAE/g) followed by curry leaves (21.94 ± 0.19 *μ*g GAE/g). Nutmeg had the lowest total phenolic content (0.80 ± 0.03 *μ*g GAE/g). Some of these herbs were also evaluated for the total phenolic content in a study by Przygodzka et al. [30], namely, cardamom, cloves, coriander, nutmeg, and star anise. However, the values which were obtained in this study were much higher, most likely owing to the method of extraction as well as the source from which they were obtained. In the instance of cumin, the reported total phenolic contents differed from the study by Vallverdú-Queralt et al. [31], in which the value was higher. Vallverdú-Queralt et al. [31] had also used an extraction method which differed from the present study. Overall, the extraction method and the source from where the spices were obtained have a significant effect on the final reported value as highlighted by Zheng and Wang [32]. Following the gastric phase of digestion, all spice extracts had statistically significant increases (*P* < 0.05) in the total phenolic content. The trend continued onto the duodenal phase of digestion as well (*P* < 0.05). The antioxidant activity values are shown in Tables 2 and 3. Despite the increases in the total phenolic contents in both pancreatic and duodenal digestion phases, the ORAC_FL_, ABTS, DPPH, and FRAP results did not indicate similar trends with a few exceptions. Overall, the antioxidant activity values coming from these assays were observed to have either been maintained during the digestion phases or statistically significantly increased (*P* < 0.05). The ORAC_oil_ values did not display any statistically significant increases or decreases as compared with the values prior to the gastric and duodenal digestion phases as well, with the only exception being cardamom, where a statistically significant increase (*P* < 0.05) was observed in the duodenal digestion phase. Despite the ABTS, DPPH, and FRAP assay values following an almost similar trend as the ORAC_FL_ values, their correlation with the total phenolic contents was comparatively less than the ORAC_FL_ values. A clear correlation between the TAC values was also not observed. The ORAC_FL_ assay has been applied extensively to evaluate the antioxidant capacity of a large variety of food products and many supplement and functional food companies compare their products, including juices, favorably to fruits and vegetables using the ORAC_FL_ results from those studies [15]. The ORAC_FL_ method is the currently most widely recognized assay used by food manufacturers despite its significant internal variability. From this assay, the antioxidant activity is determined using the area under the curve of a measurement of the protection from oxidation by free radicals generated in a temperature-dependent reaction. On the basis of technical issues related to temperature gradients across the plate in commonly used plate readers, this assay can have significant internal variability [30]. Although this technical issue does not pertain to end point determinations such as ABTS, FRAP, and DPPH assays, the ORAC_FL_ assay data was still included in this study for the overall determination of the TAC of the plant extracts. As a whole, it is important to run multiple antioxidant assays rather than just one method alone to get a better estimate of the antioxidant capacity of a food material. As for the ORAC_oil_ values, the measurement refers to the amount of antioxidant activity originating from lipid-soluble antioxidant compounds. From the absence of statistically significant fluctuations in the spice extracts prior to digestion, it may be concluded that the lipid-soluble antioxidant compounds are relatively stable against the chemical and enzymatic reactions taking place in the gastric and duodenal digestion phases as compared with the water-soluble antioxidant compounds.

Changes to the total monomeric anthocyanin content and the individual anthocyanin compounds are shown in Tables 4 and 5, respectively. Changes to the carotenoid contents are shown in Table 6. While the anthocyanin contents had statistically significant decreases (*P* > 0.05) for all the compounds analyzed, this was in contrast to the carotenoid contents where they were not observed to have statistically significant changes following gastric and duodenal digestion. It could be highlighted in this instance that the statistically significant decrease (*P* > 0.05) observed in the anthocyanin contents does not necessarily indicate a reduction in the amount of compounds. Structural transformation of the anthocyanins, especially under the varied pH conditions of the digestion model, would render them undetectable by the total monomeric and HPLC-based methods employed for the analysis. This conclusion was further supported by the analysis of total phenolic contents in Table 1. Assessment of the anthocyanin contents was essential given that spices and herbs are known to contain copious amounts of these compounds, resulting in the flavor and colour they are known to impart in food products. Given their therapeutic properties, assessment of the bioavailability of these compounds during physiological digestion could be deemed as vital. Nevertheless, the chemical structure of anthocyanins does deem them more vulnerable to ring fission, resulting in somewhat of a loss of their therapeutic effects [14]. The carotenoids which were selected for quantification in this study were based on previous evidence as to their therapeutic effects [33–36]. Nevertheless, carotenoids as an entire group of compounds could be deemed as being more relatively stable as compared with phenolic compounds when it comes to exposure to gastric and duodenal digestion conditions.

Overall, in terms of the antioxidant capacity and associated therapeutic compounds, the results showed the antioxidant capacity of the spice extracts was stable during gastric and duodenal digestion. In the study by Bermúdez-Soto et al. [37], the researchers reported a reduction in various polyphenols following similar two phase digestions of a variety of fruit juices, where a largely increased polyphenol content was shown after the gastric phase; however, these contents fell below the predigestion levels after the duodenal phase. In this instance as well, it may be hypothesized that this may have been due to a structural transformation in the polyphenols which render them undetectable by HPLC—a hypothesis which was brought forward in the study by Wootton-Beard et al. [7] as well. However, Bermúdez-Soto et al. [37] had not quantified the total phenolic content—an aspect which would have provided a better idea as to confirmation of the hypotheses. In addition, in comparison with the study by Bermúdez-Soto et al. [37], this research work also highlights the efficacy of multiple methods of analysis to prevent the exaggerated reporting of the antioxidant potential of plant-based food products.

### 3.2. Starch Hydrolase Inhibitory Activities

Inhibition of starch hydrolases could be deemed as a more novel aspect when it comes to the properties of functional food. This inhibitory activity leads to a reduced breakdown of glucose, thereby controlling the amount of calories and insulin response in a physiological system. The starch hydrolase inhibitory activities of the spice extracts are shown in Table 7. With the exception of the cumin seed extract, none of the spice extracts showed statistically significant changes to the initial enzyme inhibitory values prior to gastric and duodenal digestion. This observation was of therapeutic significance, given that the initial starch hydrolase inhibitory activities of the spice extracts were maintained despite the digestion reactions. Fenugreek had the highest *α*-amylase and *α*-glucosidase inhibitory activities, while cumin seeds had the lowest. Overall, the spices were observed to inhibit *α*-amylase better than *α*-glucosidase, given the mean inhibitory values. Inhibition of *α*-amylase is considered to be more important when it comes to reducing the breakdown of starch, since it triggers the production of the substrate for the subsequent action of *α*-glucosidase [38]. Therefore, it was noteworthy in terms of therapeutic significance that the spice extracts were able to inhibit *α*-amylase better than *α*-glucosidase. Given this requirement, even many of the commercially available antidiabetic drugs to date, such as acarbose, primarily target the inhibition of *α*-amylase rather than *α*-glucosidase. A clear correlation between the starch hydrolase inhibitory activities, total phenolic contents, and anthocyanins or carotenoid contents was not observed in this study. Thus, the starch hydrolase inhibitory potential may not have been necessarily drawn from the class of compounds which were investigated and quantified in this study.

## 4. Conclusions

This study was able to prove that the 10 spices were a significant source of total phenolics, antioxidant activity, and starch hydrolase inhibitory activities, despite the wide variety in the values observed from these parameters of analysis. However, the bioaccessibility and therefore the bioavailability of the compounds which impart the antioxidant properties need to be further evaluated prior to arriving at formidable conclusions as to their efficacy against disease conditions. With the design chosen, the study simply evaluated how the digestion process affects phenolic compounds and carotenoids already extracted, but during the real digestion process, these components may interact with other food constituents, affecting the overall bioaccessibility of the bioactive compounds. Nevertheless, this study was able to provide the first measurement concerning the stability of the antioxidant and starch hydrolase inhibitory potential of these particular spices following* in vitro* digestion. Although cell-based, animal-based, or clinical trial-based studies are able to provide more conclusive evidence, the* in vitro* digestion model used in this study could be used as a preliminary screening step prior to embarking on study models which require much more resources and planning. The study also emphasizes the importance of using multiple methods of analysis for the measurement of the total antioxidant capacity in the absence of any single accepted assay. The importance of this practice has been further highlighted in the study by Wootton-Beard et al. [7] as well as Wootton-Beard and Ryan [39], thus justifying the usage of multiple methods in this study as well.

## Figures and Tables

**Table 1:** Total phenolic content of the spices prior to digestion as well as after gastric and duodenal digestion. ^*∗*^ *P* < 0.05 denotes statistically significant difference as compared with the respective values prior to *in vitro* digestion. Values represent mean ± SEM of 3 ≤ independent experiments.

Spice	Prior (*µ*g GAE/g)	Gastric (*µ*g GAE/g)	Duodenal (*µ*g GAE/g)
Cloves	22.83 ± 0.20	23.20 ± 0.03^*∗*^	23.25 ± 0.02^*∗*^
Curry leaves	21.94 ± 0.19	23.87 ± 0.02^*∗*^	23.89 ± 0.01^*∗*^
Sweet cumin	4.99 ± 0.19	5.301 ± 0.14^*∗*^	5.312 ± 0.03^*∗*^
Cumin seeds	4.92 ± 0.07	5.29 ± 0.17^*∗*^	5.48 ± 0.03^*∗*^
Coriander	4.23 ± 0.12	5.16 ± 0.02^*∗*^	5.24 ± 0.04^*∗*^
Mustard	3.76 ± 0.04	4.092 ± 0.16^*∗*^	4.47 ± 0.20^*∗*^
Fenugreek	3.56 ± 0.03	4.66 ± 0.24^*∗*^	4.82 ± 0.03^*∗*^
Star anise	3.25 ± 0.13	4.13 ± 0.06^*∗*^	4.25 ± 0.04^*∗*^
Cardamom	1.18 ± 0.06	1.86 ± 0.08^*∗*^	1.87 ± 0.04^*∗*^
Nutmeg	0.80 ± 0.03	0.90 ± 0.06^*∗*^	0.92 ± 0.04^*∗*^

**Table 2:** Changes to the ORAC_FL_ and ORAC_oil_ values in *µ*mol Trolox Equivalents per gram (*µ*mol TE/g) of the spices prior to digestion as well as after gastric and duodenal digestion. ^*∗*^ *P* < 0.05 denotes statistically significant difference as compared with the respective values prior to *in vitro *digestion. Values represent mean ± SEM of 3 ≤ independent experiments.

Spice	ORAC_FL_ (*µ*mol TE/g)			ORAC_oil_ (*µ*mol TE/g)		
	Prior	Gastric	Duodenal	Prior	Gastric	Duodenal
Cloves	782.1 ± 6.5	785.6 ± 2.5	724.9 ± 1.1	658.2 ± 4.7	649.8 ± 3.9	658.9 ± 3.8
Curry leaves	752.6 ± 4.8	755.9 ± 2.1^*∗*^	758.9 ± 1.6	642.9 ± 3.8	641.9 ± 3.7	647.9 ± 2.5
Sweet cumin	238.9 ± 5.8	231.2 ± 1.9	237.8 ± 2.1^*∗*^	542.1 ± 2.9	539.8 ± 2.7	548.1 ± 3.1
Cumin seeds	210.3 ± 3.5	231.2 ± 1.9^*∗*^	229.8 ± 2.1^*∗*^	489.6 ± 6.5	479.6 ± 5.8	487.1 ± 2.4
Coriander	197.5 ± 3.2	185.9 ± 1.3^*∗*^	189.7 ± 1.4^*∗*^	471.8 ± 3.9	467.8 ± 3.8	467.5 ± 2.1
Mustard	177.5 ± 2.3	180.3 ± 1.6	185.9 ± 2.3	408.9 ± 5.4	410.8 ± 2.7	411.2 ± 3.7
Fenugreek	165.2 ± 3.4	165.9 ± 1.4	167.5 ± 1.6	359.8 ± 2.8	361.7 ± 2.4	357.6 ± 4.7
Star anise	158.4 ± 2.6	159.7 ± 1.5	159.3 ± 1.2	347.2 ± 3.9	359.2 ± 3.4	359.2 ± 3.7
Cardamom	92.5 ± 3.5	89.7 ± 2.0^*∗*^	91.2 ± 1.3^*∗*^	318.7 ± 2.6	320.6 ± 2.5	342.0 ± 1.9^*∗*^
Nutmeg	65.8 ± 1.2	63.8 ± 1.8^*∗*^	75.4 ± 1.8^*∗*^	304.9 ± 2.1	305.1 ± 2.8	306.4 ± 2.9

**Table 3:** Changes to the ABTS, DPPH, and FRAP assay values of the spices prior to digestion as well as after gastric and duodenal digestion. ^*∗*^ *P* < 0.05 denotes statistically significant difference as compared with the respective values prior to *in vitro *digestion. Values represent mean ± SEM of 3 ≤ independent experiments.

Spice	ABTS (*µ*mol TE/g)			DPPH (EC_50_, mg/kg)			FRAP (*µ*mol TE/g)		
	Prior	Gastric	Duodenal	Prior	Gastric	Duodenal	Prior	Gastric	Duodenal
Cloves	198.7 ± 1.9	195.9 ± 2.4	197.2 ± 1.7	65.8 ± 2.5	67.8 ± 1.9	67.8 ± 2.7	2698 ± 10	2254 ± 19^*∗*^	2257 ± 11^*∗*^
Curry leaves	182.4 ± 3.6	182.4 ± 1.9	185.8 ± 1.4	69.8 ± 1.8	64.8 ± 1.6	69.8 ± 2.4	2158 ± 11	2125 ± 14	2124 ± 16
Sweet cumin	163.5 ± 2.4	168.9 ± 1.7	162.4 ± 1.4	75.4 ± 1.9	78.7 ± 4.5	74.9 ± 4.7	1759 ± 21	1758 ± 21	1747 ± 14
Cumin seeds	152.4 ± 1.9	152.0 ± 3.1	155.9 ± 1.5	84.1 ± 1.7	88.5 ± 1.4^*∗*^	89.6 ± 1.7^*∗*^	1542 ± 14	1525 ± 20	1547 ± 19
Coriander	144.2 ± 3.1	148.9 ± 1.7	149.5 ± 1.8	91.4 ± 2.5	97.8 ± 2.5^*∗*^	99.6 ± 2.8^*∗*^	1420 ± 13	1458 ± 14	1447 ± 21
Mustard	124.7 ± 1.8	125.4 ± 1.1	122.5 ± 1.5	110.2 ± 3.4	115.9 ± 2.4	112.8 ± 1.5	1025 ± 17	1014 ± 10	1189 ± 17^*∗*^
Fenugreek	114.7 ± 1.9	113.2 ± 1.4	112.0 ± 1.9	127.4 ± 2.5	128.9 ± 1.7	124.2 ± 1.4	1022 ± 12	932 ± 10^*∗*^	1055 ± 19
Star anise	92.5 ± 4.3	91.6 ± 1.8	91.8 ± 1.4	178.4 ± 2.9	177.2 ± 1.8	178.9 ± 2.4	954 ± 16	947 ± 14	957 ± 10
Cardamom	64.2 ± 1.9	65.6 ± 1.8	52.9 ± 1.1^*∗*^	188.7 ± 1.8	187.4 ± 2.4	188.9 ± 2.3	847 ± 10	841 ± 11	858 ± 17
Nutmeg	52.8 ± 1.4	53.9 ± 1.8	51.4 ± 1.1	197.5 ± 4.5	199.8 ± 4.7	189.5 ± 4.8	721 ± 16	754 ± 19	759 ± 14

**Table 4:** The total monomeric anthocyanin pigment contents of the spices prior to digestion as well as after gastric and duodenal digestion in mg cyaniding-3-glucoside equivalents per g wet weight of spice (mg/g). ^*∗*^ *P* < 0.05 denotes statistically significant difference as compared with the respective values prior to *in vitro *digestion. Values represent mean ± SEM of 3 ≤ independent experiments.

Spice	Prior (mg/g)	Gastric (mg/g)	Duodenal (mg/g)
Cloves	89.8 ± 2.5	59.2 ± 6.5^*∗*^	56.8 ± 1.6^*∗*^
Curry leaves	58.9 ± 1.8	29.8 ± 1.9^*∗*^	31.5 ± 2.4^*∗*^
Sweet cumin	48.3 ± 1.6	26.5 ± 1.2^*∗*^	29.8 ± 3.5^*∗*^
Cumin seeds	48.7 ± 2.0	25.6 ± 1.3^*∗*^	26.8 ± 1.9^*∗*^
Coriander	35.9 ± 2.5	20.8 ± 1.4^*∗*^	19.8 ± 2.1^*∗*^
Mustard	30.2 ± 2.0	19.6 ± 2.1^*∗*^	19.2 ± 1.0^*∗*^
Fenugreek	31.2 ± 1.8	18.9 ± 1.9^*∗*^	18.2 ± 1.5^*∗*^
Star anise	28.5 ± 1.2	19.6 ± 1.1^*∗*^	18.9 ± 1.5^*∗*^
Cardamom	27.5 ± 1.1	18.5 ± 1.2^*∗*^	17.9 ± 1.6^*∗*^
Nutmeg	26.3 ± 1.4	15.2 ± 1.1^*∗*^	14.9 ± 1.8^*∗*^

**Table 5:** Quantities of D3Ga, C3Ga, C3Gl, C3Ar, P3Ga, and P3Ar present in the herbal extracts prior to digestion (P) as well as after gastric (G) and duodenal (D) digestion. ^*∗*^ *P* < 0.05 denotes statistically significant difference as compared with prior *in vitro* digestion. Values represent mean ± SEM of 3 ≤ independent experiments.

Spice	D3Ga (mg/g)			C3Ga (mg/g)			C3GI (mg/g)			C3Ar (mg/g)			P3Ga (mg/g)			P3Ar (mg/g)		
	P	G	D	P	G	D	P	G	D	P	G	D	P	G	D	P	G	D
Cloves	1.21 ± 0.09	0.50 ± 0.08^*∗*^	0.27 ± 0.01^*∗*^	1.80 ± 0.08	1.00 ± 0.07^*∗*^	0.98 ± 0.06^*∗*^	2.10 ± 0.06	1.25 ± 0.08^*∗*^	1.15 ± 0.05^*∗*^	1.39 ± 0.04	0.68 ± 0.08^*∗*^	0.58 ± 0.01^*∗*^	1.95 ± 0.01	1.47 ± 0.02^*∗*^	1.17 ± 0.04^*∗*^	1.67 ± 0.02	1.24 ± 0.03^*∗*^	1.15 ± 0.01^*∗*^
Curry leaves	0.98 ± 0.02	0.74 ± 0.10^*∗*^	0.69 ± 0.08^*∗*^	1.44 ± 0.09	1.22 ± 0.04^*∗*^	0.54 ± 1.47^*∗*^	1.21 ± 0.08	1.22 ± 0.06^*∗*^	0.88 ± 0.04^*∗*^	0.66 ± 0.04	0.58 ± 0.01^*∗*^	0.47 ± 0.04^*∗*^	0.87 ± 0.02	0.74 ± 0.01^*∗*^	0.69 ± 0.02^*∗*^	1.21 ± 0.04	0.89 ± 0.10^*∗*^	0.63 ± 0.05^*∗*^
Sweet cumin	0.47 ± 0.01	0.23 ± 0.01^*∗*^	0.19 ± 0.02^*∗*^	0.49 ± 0.04	0.39 ± 0.07^*∗*^	0.22 ± 0.04^*∗*^	1.24 ± 0.02	1.00 ± 0.04^*∗*^	0.95 ± 0.11^*∗*^	0.95 ± 0.08	0.67 ± 0.05^*∗*^	0.62 ± 0.02^*∗*^	1.49 ± 0.09	0.25 ± 0.01^*∗*^	0.31 ± 0.02^*∗*^	1.22 ± 0.07	1.20 ± 0.08^*∗*^	1.17 ± 0.04^*∗*^
Cumin seeds	1.31 ± 0.05	1.20 ± 0.01^*∗*^	1.05 ± 0.06^*∗*^	1.20 ± 0.36	0.58 ± 0.01^*∗*^	0.44 ± 0.03^*∗*^	1.35 ± 0.02	0.94 ± 0.06^*∗*^	0.84 ± 0.03^*∗*^	1.24 ± 0.06	1.15 ± 0.06^*∗*^	0.84 ± 0.05^*∗*^	0.87 ± 0.03	0.64 ± 0.02^*∗*^	0.54 ± 0.01^*∗*^	0.97 ± 0.08	0.87 ± 0.01^*∗*^	0.68 ± 0.02^*∗*^
Coriander	1.12 ± 0.05	1.00 ± 0.03^*∗*^	0.85 ± 0.02^*∗*^	0.65 ± 0.02	0.51 ± 0.02^*∗*^	0.48 ± 0.01^*∗*^	0.75 ± 0.04	0.61 ± 0.02^*∗*^	0.57 ± 0.01^*∗*^	0.67 ± 0.01	0.44 ± 0.02^*∗*^	0.42 ± 0.01^*∗*^	0.74 ± 0.01	0.59 ± 0.01^*∗*^	0.54 ± 0.02^*∗*^	0.64 ± 0.02	0.29 ± 0.01^*∗*^	0.22 ± 0.02^*∗*^
Mustard	0.58 ± 0.02	0.25 ± 0.01^*∗*^	0.20 ± 0.01^*∗*^	0.67 ± 0.02	0.61 ± 0.03^*∗*^	0.54 ± 0.08^*∗*^	0.81 ± 0.03	0.61 ± 0.02^*∗*^	0.51 ± 0.04^*∗*^	0.74 ± 0.01	0.61 ± 0.03^*∗*^	0.51 ± 0.02^*∗*^	0.94 ± 0.01	0.88 ± 0.04^*∗*^	0.77 ± 0.02^*∗*^	0.47 ± 0.02	0.36 ± 0.07^*∗*^	0.29 ± 0.01^*∗*^
Fenugreek	0.39 ± 0.02	0.11 ± 0.01^*∗*^	0.10 ± 0.01^*∗*^	0.48 ± 0.03	0.32 ± 0.02^*∗*^	0.25 ± 0.01^*∗*^	0.55 ± 0.04	0.51 ± 0.03^*∗*^	0.50 ± 0.03^*∗*^	0.47 ± 0.06	0.31 ± 0.03^*∗*^	0.31 ± 0.01^*∗*^	0.77 ± 0.03	0.65 ± 0.04^*∗*^	0.54 ± 0.01^*∗*^	0.66 ± 0.02	0.60 ± 0.01^*∗*^	0.54 ± 0.02^*∗*^
Star anise	0.85 ± 0.02	0.65 ± 0.01^*∗*^	0.60 ± 0.02^*∗*^	0.80 ± 0.01	0.75 ± 0.02^*∗*^	0.75 ± 0.01^*∗*^	0.66 ± 0.05	0.49 ± 0.01^*∗*^	0.45 ± 0.02^*∗*^	0.58 ± 0.02	0.55 ± 0.05^*∗*^	0.50 ± 0.03^*∗*^	0.49 ± 0.01	0.39 ± 0.02^*∗*^	0.28 ± 0.01^*∗*^	0.33 ± 0.02	0.28 ± 0.05^*∗*^	0.25 ± 0.01^*∗*^
Cardamom	0.79 ± 0.01	0.52 ± 0.01^*∗*^	0.49 ± 0.01^*∗*^	0.38 ± 0.02	0.31 ± 0.01^*∗*^	0.29 ± 0.02^*∗*^	0.84 ± 0.02	0.77 ± 0.03^*∗*^	0.75 ± 0.02^*∗*^	0.29 ± 0.01	0.25 ± 0.02^*∗*^	0.25 ± 0.01^*∗*^	0.36 ± 0.04	0.32 ± 0.02^*∗*^	0.31 ± 0.01^*∗*^	0.68 ± 0.02	0.62 ± 0.05^*∗*^	0.60 ± 0.03^*∗*^
Nutmeg	0.57 ± 0.02	0.41 ± 0.01^*∗*^	0.40 ± 0.04^*∗*^	0.87 ± 0.05	0.81 ± 0.06^*∗*^	0.74 ± 0.06^*∗*^	0.91 ± 0.06	0.72 ± 0.03^*∗*^	0.61 ± 0.05^*∗*^	0.88 ± 0.04	0.71 ± 0.06^*∗*^	0.66 ± 0.05^*∗*^	0.49 ± 0.01	0.34 ± 0.02^*∗*^	0.30 ± 0.02^*∗*^	0.45 ± 0.02	0.26 ± 0.01^*∗*^	0.26 ± 0.01^*∗*^

**Table 6:** Quantities of neoxanthin, violaxanthin, lutein, zeaxanthin, *α*-carotene, and  *β*-carotene present in the herbal extracts prior to digestion (P) as well as after gastric (G) and duodenal (D) digestion. *P* < 0.05 denotes statistically significant difference as compared with the respective values prior to *in vitro *digestion. Values represent mean ± SEM of 3 ≤ independent experiments.

Spice	Neoxanthin (mg/g)			Violaxanthin (mg/g)			Lutein (mg/g)			Zeaxanthin (mg/g)			*α*-Carotene (mg/g)			*β*-Carotene (mg/g)		
	P	G	D	P	G	D	P	G	D	P	G	D	P	G	D	P	G	D
Cloves	0.78 ± 0.05	0.75 ± 0.06	0.77 ± 0.02	1.10 ± 0.08	1.11 ± 0.09	1.15 ± 0.08	1.15 ± 0.09	1.12 ± 0.05	1.13 ± 0.02	0.95 ± 0.08	0.96 ± 0.08	0.97 ± 0.08	1.28 ± 0.01	1.29 ± 0.02	1.29 ± 0.02	1.28 ± 0.01	1.25 ± 0.02	1.26 ± 0.02
Curry leaves	0.62 ± 0.05	0.65 ± 0.04	0.66 ± 0.03	0.87 ± 0.02	0.88 ± 0.03	0.89 ± 0.05	0.79 ± 0.02	0.78 ± 0.03	0.79 ± 0.02	1.18 ± 0.02	1.17 ± 0.03	1.15 ± 0.06	0.84 ± 0.02	0.84 ± 0.02	0.85 ± 0.01	0.79 ± 0.05	0.80 ± 0.04	0.81 ± 0.02
Sweet cumin	0.79 ± 0.01	0.81 ± 0.02	0.80 ± 0.01	1.08 ± 0.09	1.09 ± 0.02	1.09 ± 0.02	0.88 ± 0.02	0.87 ± 0.01	0.87 ± 0.01	0.88 ± 0.06	0.87 ± 0.05	0.88 ± 0.06	1.05 ± 0.06	1.05 ± 0.03	1.04 ± 0.06	0.95 ± 0.06	0.95 ± 0.05	0.95 ± 0.04
Cumin seeds	1.10 ± 0.03	1.12 ± 0.01	1.12 ± 0.02	0.55 ± 0.01	0.56 ± 0.02	0.56 ± 0.01	0.62 ± 0.01	0.63 ± 0.01	0.63 ± 0.01	0.58 ± 0.02	0.56 ± 0.01	0.55 ± 0.02	0.49 ± 0.01	0.48 ± 0.01	0.48 ± 0.01	0.64 ± 0.09	0.66 ± 0.05	0.65 ± 0.01
Coriander	0.65 ± 0.01	0.69 ± 0.04	0.69 ± 0.04	0.75 ± 0.01	0.76 ± 0.02	0.76 ± 0.01	0.85 ± 0.02	0.86 ± 0.01	0.86 ± 0.01	0.69 ± 0.01	0.70 ± 0.02	0.70 ± 0.02	0.65 ± 0.01	0.66 ± 0.02	0.66 ± 0.01	0.59 ± 0.03	0.59 ± 0.01	0.59 ± 0.01
Mustard	0.84 ± 0.03	0.85 ± 0.01	0.85 ± 0.01	0.71 ± 0.02	0.70 ± 0.02	0.70 ± 0.02	0.66 ± 0.01	0.66 ± 0.01	0.66 ± 0.01	0.59 ± 0.01	0.59 ± 0.01	0.58 ± 0.02	0.61 ± 0.02	0.61 ± 0.02	0.61 ± 0.02	0.63 ± 0.09	0.65 ± 0.01	0.65 ± 0.02
Fenugreek	0.45 ± 0.01	0.46 ± 0.01	0.46 ± 0.01	0.58 ± 0.02	0.58 ± 0.01	0.58 ± 0.01	0.62 ± 0.01	0.62 ± 0.02	0.62 ± 0.02	0.39 ± 0.02	0.40 ± 0.01	0.40 ± 0.01	0.49 ± 0.01	0.48 ± 0.01	0.48 ± 0.01	0.61 ± 0.02	0.62 ± 0.02	0.62 ± 0.02
Star anise	0.39 ± 0.03	0.39 ± 0.02	0.40 ± 0.02	0.88 ± 0.03	0.85 ± 0.04	0.86 ± 0.05	0.90 ± 0.02	0.91 ± 0.01	0.90 ± 0.04	0.62 ± 0.03	0.61 ± 0.09	0.61 ± 0.08	0.69 ± 0.08	0.70 ± 0.07	0.71 ± 0.06	0.61 ± 0.03	0.61 ± 0.02	0.61 ± 0.01
Cardamom	0.35 ± 0.02	0.36 ± 0.02	0.36 ± 0.01	0.54 ± 0.02	0.55 ± 0.01	0.55 ± 0.01	0.62 ± 0.04	0.65 ± 0.02	0.69 ± 0.05	0.71 ± 0.02	0.71 ± 0.02	0.71 ± 0.02	0.69 ± 0.01	0.69 ± 0.01	0.69 ± 0.01	0.53 ± 0.04	0.53 ± 0.04	0.53 ± 0.02
Nutmeg	0.39 ± 0.01	0.41 ± 0.02	0.41 ± 0.02	0.51 ± 0.03	0.55 ± 0.01	0.55 ± 0.01	0.49 ± 0.01	0.48 ± 0.02	0.48 ± 0.01	0.66 ± 0.02	0.66 ± 0.01	0.65 ± 0.01	0.71 ± 0.02	0.71 ± 0.02	0.72 ± 0.02	0.31 ± 0.05	0.31 ± 0.05	0.30 ± 0.01

**Table 7:** *α*-Amylase and *α*-glucosidase inhibitory activities of the spice extracts prior and following digestion in the gastric and duodenal phases. ^*∗*^ *P* < 0.05 denotes statistically significant difference as compared with the respective values prior to *in vitro *digestion.

Sample code	*α*-Amylase inhibitory activity			*α*-Glucosidase inhibitory activity		
	Prior (IC_50_, *μ*g/mL)	Gastric (IC_50_, *μ*g/mL)	Duodenal (IC_50_, *μ*g/mL)	Prior (IC_50_, *μ*g/mL)	Gastric (IC_50_, *μ*g/mL)	Duodenal (IC_50_, *μ*g/mL)
Fenugreek	48.9 ± 1.6	49.5 ± 3.6	48.9 ± 1.8	55.8 ± 1.9	56.7 ± 1.4	56.9 ± 1.7
Curry leaves	55.9 ± 1.4	58.7 ± 1.9	58.9 ± 1.8	59.6 ± 1.5	60.2 ± 1.6	61.2 ± 1.8
Coriander	60.3 ± 1.8	61.4 ± 1.8	61.9 ± 1.7	69.8 ± 1.4	70.8± 1.6	71.9 ± 1.4
Nutmeg	75.9 ± 1.2	75.9 ± 1.2	76.8 ± 1.9	81.2 ± 1.7	82.6 ± 1.6	83.9 ± 1.4
Star anise	83.6 ± 1.6	84.9 ± 1.5	88.7 ± 1.4	92.6 ± 1.9	95.8 ± 2.0	96.8 ± 2.1
Sweet cumin	104.9 ± 1.9	106.2 ± 1.7	109.5 ± 2.1	119.5 ± 1.1	120.3 ± 1.2	121.5 ± 1.8
Cloves	128.9 ± 3.6	139.5 ± 2.4^*∗*^	140.2 ± 3.6^*∗*^	149.8 ± 2.6	151.9 ± 2.4	154.3 ± 2.5
Mustard	169.8 ± 2.6	170.6 ± 2.8	171.6 ± 2.4	179.6 ± 1.5	184.6 ± 2.1	188.4 ± 2.6
Cardamom	197.9 ± 1.6	198.6 ± 1.7	198.6 ± 1.7	256.3 ± 6.4	256.9 ± 6.2	256.9 ± 6.2
Cumin seeds	254.6 ± 4.8	269.4 ± 4.8^*∗*^	266.1 ± 4.7^*∗*^	279.6 ± 2.6	281.6 ± 2.5	281.4 ± 2.3
